# Antioxidant Indexes and Immune Function of the Intestinal Flora of Compound Microecological Preparations

**DOI:** 10.1155/2022/5498514

**Published:** 2022-09-30

**Authors:** Wanzhen Sun, Li Zhang

**Affiliations:** ^1^Clinical Laboratory, Wuhan Mental Health Center, Wuhan, 430012 Hubei Province, China; ^2^Clinical Laboratory, The Second Staff Hospital of Wuhan Iron and Steel (Group) Company, Wuhan, 430085 Hubei, China

## Abstract

Compound probiotics are biological products made by mixing and cultivating various probiotics according to appropriate composition and ratio. It can not only play the role of a variety of probiotics in composition but also the effect of the ratio is often greater than the effect of the single strain alone. These probiotics are good for the body's immune system in living organisms. They act as immune boosters in living organisms. They are considered the safest form of treatment. In this review, the effects of microecological agents on antioxidant indices and immune function of chicks were studied, and radial basis neural network (RBFNN) was described. Aiming at the deficiency of traditional RBFNN learning strategy, a three-layer RBFNN method based on immune mechanism was proposed. In this paper, the microecological evaluation preparation was added into chicken feed. The study showed that chickens fed with probiotics gained significant body weight at 6 weeks of age. Compared with the control group, the experimental group increased by 15.70%. In each feed/gain ratio, the feed/gain ratio of the experimental group was significantly decreased at 6 weeks of age, which was 30.37% lower than that of the control group. Compared with the control group, the spleen, bursa of Fabricius, and thymus of the experimental group were increased by 63.02%, 38.77%, and 26.82%, respectively, indicating that the compound probiotics could improve the immunity of chickens.

## 1. Introduction

Compound microecological preparations can help the body return to normal nutrition, growth, and health, and it is one of the more popular new feed additives in current research. Adding it to animal diets can achieve an effect similar to antibiotics to a certain extent. Because of its green, nontoxic, nondrug-resistant, safe, and efficient characteristics, it has been gradually used in the livestock breeding industry. For example, poultry farming plays an important role in developing China's animal husbandry and is the world's second-largest poultry producer and consumer. On the other hand, most microecological products currently on the market are composed of one or more lactic acid bacteria, bacilli, and yeasts of the same genus. While the microecological preparations composed of different genus microorganisms can play their respective advantages, they can also compensate for the insufficiency of a single strain. Therefore, it has gradually become the trend of research and development of compound microecological preparations and has achieved good use effects and considerable economic benefits. Among living things, these probiotics are excellent for the immune system of the body. They strengthen the immune systems of living things. Therefore, they are regarded as the most secure form of therapy.

The growing number of studies investigating the use of review probiotics to improve patient health outcomes has prompted the need for a systematic review and summary of the relevant literature. Wang et al. summarized the origin and characteristics of Chinese medicine-probiotic mixed livestock and poultry microecological preparations (CPCMP) strain based on reviewing the literature on probiotics and traditional Chinese medicine microecological preparations in recent years [1]. Given the complex composition of traditional Chinese medicine compound preparations and the unclear mechanism of action which restricts the development of traditional Chinese medicine, Jie et al. has achieved extensive and remarkable results [2]. Naito et al. used compound-specific stable isotope analysis of amino acids (CSIA) to study terrestrial mammals in a controlled feeding experiment of captive Asian black bears [3]. Guo et al. studied the etiology, characteristics, and relatively effective treatment methods of three common gastrointestinal diseases, including diarrhea, constipation, and irritable bowel syndrome, based on gut microbes. Taking diarrhea, constipation, and irritable bowel syndrome as examples, the role and mechanism of traditional Chinese medicine and microecological substances in gastrointestinal diseases were discussed to provide a reference for more reasonable and effective treatment of gastrointestinal diseases [4]. The Kokaeva et al. study aimed at developing a method to improve the ecological and consumption characteristics of dairy cows and their derived milk by rationally using antioxidant toxins and mold Zap in diets containing subtoxic doses of nitrate and aflatoxin B1 [5]. However, the impact of reviewing microecological preparations needs to be examined from multiple perspectives to be more comprehensive.

Artificial intelligence is an important technical tool to support the development of information fusion, among which RBFNN is another hot spot of intelligence research. For problems involving function approximation, radial basis function (RBF) networks are a popular variety of artificial neural networks. The universal approximation and quicker learning speed of radial basis function networks set them apart from other neural networks. Moreira et al. proposed the modeling, performance evaluation, and comparative analysis of an artificial neural network technique called Radial Basis Function Network (RBFNN network) to identify gestational diabetes cases that may lead to multiple risks to the mother and fetus [6]. Leema et al. discussed a classification framework for diagnosing diseases using a Quantum Behavioral Particle Swarm Optimization Neural Network (QPSONN) classifier, and the neural network used for classification is RBFNN [7]. Amin et al. proposed an ENRBFN that approximates the unmodeled dynamics of a hovering vehicle based on an adaptive trajectory tracking controller based on the Extended Normalized Radial Basis Function (ENRBF) [8]. Mohapatra and Mohanty described how the demand for hospital services is increasing daily, and intelligent services for patients are critical to calculating mortality rates. A method for detecting arrhythmias using wavelet transform and data mining techniques was adopted [9]. Pomprapa et al. proposed the application of backstepping control in the oxygenation of the cardiopulmonary system. Without prior knowledge of the underlying system dynamics, an RBF network was integrated into a closed-loop subsystem and trained to recognize unknown nonlinear functions [10]. These algorithms achieve the research goals to a certain extent, but the rationality of the calculation process can be further improved. The compound probiotic microecological preparation was applied to the chicks. By measuring the weight gain, feed-to-weight ratio and immune organs, and other indices of the chickens, it was found that the compound probiotic microecological preparation promoted growth and had a positive effect on the immune function of chickens. The innovation of this paper is that through the experimental study of chicken activity, compound probiotics are added to chicken feed to improve chicken growth performance, feed utilization rate, and immunity. In every capsule of the probiotic complex, there are 6 billion friendly bacteria. These bacteria include Lactobacillus acidophilus, which typically colonizes the upper intestine, and Bifidobacterium bifidum, which typically colonizes the lower intestine. The ability of these bacteria to produce lactic acid as a byproduct of glucose metabolism distinguishes them from other bacteria. Gram-positive bacteria, such as Lactobacillus, are defined as having a thick peptidoglycan cell wall.

The rest of the paper is organized as section 2 gives RBFNN method based on the immune system, section 3 gives an experiment on the effect of compound microecological preparation on chicks, section 4 gives us results, and the conclusion is given in section 5.

## 2. RBFNN Method Based on Immune System

In this section, we will discuss the biological immune system, RBF network learning strategy, and design of RBF NN based on the immune system in detail.

### 2.1. Biological Immune System

The immune system protects the body from pathogens through a multilayered defense structure, and as the defense layer increases, its specificity for pathogens increases layer by layer. An organism that infects its host with the disease is referred to as a pathogen, and the severity of the disease symptoms is referred to as virulence. Pathogens include viruses, bacteria, unicellular, and multicellular eukaryotes, as well as other taxonomically diverse organisms. Briefly, this hierarchical structure is divided into three lines of defense, which can be classified into two categories: innate immunity and specific immunity [11, 12], as shown in Figure 1.

This part mainly introduces the biological immune system mechanism related to the proposed algorithm, and readers can refer to other aspects of the mechanism. The biological immune system is composed of many complex cells, molecules, and organs. These tissues can cope with foreign virus infection to achieve the function of protecting the health and stability of the body. The biological immune system includes two related subsystems, innate immunity, and adaptive immunity. The organic combination of these two subsystems can recognize and eliminate foreign viruses, bacteria, etc., to achieve the function of defense [13]. These infectious agents are hereinafter collectively referred to as antigens.

Figure 2 is a schematic diagram of the mechanism of interaction between innate and adaptive immunity. When Ag invades the body, a specific antigen-presenting cell in the innate immune system can quickly recognize the invading Ag and absorb and decompose it into many gene segments. These decomposed gene segments are adsorbed to the cell's major histocompatibility complex (MHC) to form MHC protein receptors. The MHC is a collection of genes that produce proteins found on the cell surfaces and aid the immune system in recognizing.

Major Histocompatibility Complex (MHC) is a collection of genes that produce proteins found on the cell surfaces and aid in the immune system's ability to identify foreign objects. The higher vertebrates contain MHC proteins. The complex is also known as the human leukocyte antigen (HLA) system in humans. These receptors are presented on the surface of the MHC, and T cells in the immune system also have a receptor molecule on the surface that recognizes different MIHC complexes. Once T cells recognize the MHC complex, they are activated to secrete or differentiate into lymphocytes or other chemical signals. These cellular or chemical signals stimulate other elements of the immune system to facilitate the development of an adaptive immune response [14, 15].

Immune response, immune tolerance, and immune feedback are the three stages of the immune mechanism. After the antigen enters the body, the immune cells recognize the antigen molecule and undergo the corresponding process of cell activation, cell differentiation, and immune function, that is, an immune response. In the process of an immune response, several steps are included, such as specific recognition, antigen presentation, lymphocyte activation, antibody generation, an immune reaction between antibody and antigen, and the formation of immune memory [16]. One of the key features of the immune system is its capacity for learning and memory, which is demonstrated by the immune system's capacity to remember the antigenic structure it encounters for the first time. Antigen specificity and long-lasting effects are features of immune memory. The primary distinction between humoral and cell-mediated immunity is the production of antigen-specific antibodies by humoral immunity as opposed to cell-mediated immunity. T lymphocytes, however, obliterate infected cells. Immune feedback has two corresponding feedback mechanisms for humoral immunity and cellular immunity, and the principle is shown in Figure 3.

In Layman's terms, immunity is a physiological reflection that aims at identifying self and nonself and, at the same time, remove nonself to ensure the integrity of the body. After a fight with a pathogen (antibody), the body would retain the ability to fight against the pathogen so that when the body encounters the same pathogen again, it can quickly and effectively make defenses to protect the body from damage. Compared with the specific immune system, the innate immune system is universal and memoryless, while the latter is specificity and memory [17, 18].

The ability to learn and remember is one of the main characteristics of the immune system, which is manifested in the ability of the immune system to learn and remember the antigenic structure it encounters for the first time. Immune memory is characterized by antigen specificity and durable effects [19]. Both T cells and B cells are involved in immune memory; that is, during the immune response, both memory B cells and memory T cells are present. The formation process of immune memory cells is shown in Figure 4.

### 2.2. RBF Network Learning Strategy

RBFNN is a typical local approximation network model [20]. Given the training samples, then, the learning strategy of RBFNN should solve the following problems: first, determining the structure of the network, that is, determining the number of hidden layer nodes *h* of the network; secondly, determining the data center *v*_*o*_ and width *δ*_*o*_ of each radial basis function; finally, determining the output of the network modifies the weights *e*_*o*_ and the bias q.

In RBFNN, the nonlinear activation function of the hidden layer and the linear parameters of the output layer are updated on different “time scales”. Different layers play different roles, so different update strategies can be used. There are four commonly used learning methods for RBFNN, as shown in Figure 5.

In the fourth strategy, except that the number of network nodes *j* needs to be predetermined, the other free parameters of RBFNN are trained by performing a supervised learning process, so this learning strategy identifies the generalized form of RBFNN. This strategy is mostly implemented by the error-corrected gradient descent method (An optimization algorithm called gradient descent is frequently used to train neural networks and machine learning models. These models are trained using training data, and the cost function within gradient descent specifically serves as a barometer, gauging its accuracy with each new training set), whose form is similar to the back-propagation algorithm (BP algorithm) [21].

Let (*c*_*m*_, *a*_*m*_) represent the input data, and its corresponding expected output, and *u*_*m*_ represent the actual output of the network, then the error *r*_*m*_ of the network at time *m* is

(1) $$\begin{array}{c} r_{m}=a_{m}-u_{m}. \end{array}$$

For a parameter *μ* in a network, it is adjusted by the gradient training algorithm by

(2) $$\begin{array}{c} \mu_{m+1}=\mu_{m}-\lambda_{\mu }\frac{\partial r_{m}^{2}}{\partial \mu_{m}}. \end{array}$$

In Formula (2), *λ*_*μ*_ is an adaptive coefficient. Specifically, in the RBF network, the gradient training algorithm obtains various network parameters according to

(3) $$\begin{array}{c} \Delta v_{o,m}=v_{o,m+1}-v_{o,m}=\lambda_{v}r_{m}e_{o,m}\exp\left(-\frac{{\left\|c_{m}-v_{o,m}\right\|}^{2}}{2\delta_{o,m}^{2}}\right)\frac{\left\|c_{m}-v_{o,m}\right\|}{\delta_{o,m}^{2}},\\ \Delta \delta_{o,m}=\delta_{o,m+1}-\delta_{o,m}=\lambda_{\delta }r_{m}e_{o,m}\exp\left(-\frac{{\left\|c_{m}-v_{o,m}\right\|}^{2}}{2\delta_{o,m}^{2}}\right)\frac{\left\|c_{m}-v_{o,m}\right\|}{\delta_{o,m}^{3}},\\ \Delta e_{o,m}=e_{o,m+1}-e_{o,m}=\lambda_{e}r_{m}\exp\left(-\frac{{\left\|c_{m}-v_{o,m}\right\|}^{2}}{2\delta_{o,m}^{2}}\right),\\ \Delta q_{m}=q_{m+1}-q_{m}=\lambda_{q}r_{m}. \end{array}$$

The initial search of gradient training algorithms is usually performed from the parameter space, limiting the search region of the parameter space to a known useful region. In most cases, the gradient training method provides a convenient and feasible RBF network learning strategy.

The common disadvantage of the above methods is that the global RBF network parameters cannot be obtained by learning, and most of them need to predetermine the number *h* of network center points. In addition, except for the supervised center selection method, which obtains the remaining network parameters through the supervised learning process, the other methods focus on the training of the network center *v*_*o*_. The network expansion constant *δ*_*o*_ is predesigned or determined by the distance between the data centers, and the global optimal value cannot be guaranteed. The expansion constant has an important impact on the performance of the RBF network: if its value is too large, it means that a large number of hidden nodes are needed to fit the function with a fast-changing speed, and the basis function curve overlaps the response area more; and if its value is too small, a large number of hidden nodes are needed to fit the smoother function, which would lead to the degradation of the performance of the RBF network. Of course, there are also some learning strategies based on evolutionary methods to dynamically adjust the RBF network center, but most of them have problems like the above-mentioned problem that the optimal training value of the global network parameters cannot be obtained, which may lead to problems such as excessive algorithm complexity, long training time, and easy to fall into local minima [22, 23].

### 2.3. Design of RBFNN Based on Immune System

Because of the shortcomings and problems of the above existing RBFNN learning strategies, this paper proposes an immune system-based RBFNN design and training strategy, which introduces a unique immune system-specific vaccine extraction and inoculation mechanism, thereby simplifying the network training process and optimizing its performance.

The design goal of the RBFNN learning strategy is to determine the globally optimized RBF network parameters: *ϖ* = {*j*, *v*_*o*_, *δ*_*o*_, *e*_*o*_, *q*}. The design parameter of the nonlinear neuron in the hidden layer of the network is {*j*, *v*_*o*_, *δ*_*o*_}, and {*e*_*o*_, *q*} is the design parameter of the linear neuron in the output layer of the network (*o* = 1, ⋯, *j*).

When designing a learning strategy, it is unnecessary and highly efficient to design the global parameters *ϖ* in the same optimization space. The parameter is the key to the design of the hidden layer structure and even the entire RBF network topology. Determining this parameter first can greatly simplify the network training process. Since the network output layer is a linear neuron, therefore, as long as a reasonable hidden layer of the network is constructed and the parameter {*v*_*o*_, *δ*_*o*_} is determined, the output layer parameter {*e*_*o*_, *q*} can be determined by an efficient linear optimization method.

Because of the above two points, this paper proposes a three-level learning structure strategy of RBFNN based on the immune mechanism: dividing the global RBFNN parameter space *ϖ* into three subspaces. That is, design optimization is carried out for *ϖ*_1_ = {*j*}, *ϖ*_2_ = {*v*_*o*_, *δ*_*o*_}, and *ϖ*_3_ = {*e*_*o*_, *q*}, respectively.  Figure 6 shows the three-level learning structure framework of the RBFNN: the first level calculates *ϖ*_1_ to determine the topology of the entire RBF network, and this level is a process of extracting vaccines according to the problem to be solved; the second stage is postvaccination to determine *ϖ*_2_ to identify neurons in the hidden layers of the network, and this stage is designed using an immune algorithm. The third stage uses the least squares estimation *ϖ*_3_ to determine the output layer neurons of the network. After the three-level learning, the global RBF network parameter *ϖ* = {*ϖ*_1_, *ϖ*_2_, *ϖ*_3_} is determined, that is, a complete RBF network is constructed.

The first level: extracting the vaccine and determining the network structure.

The first level mainly calculates the number of neurons in the hidden layer of the network; that is, it calculates *ϖ*_1_ = {*j*}. Let the maximum number of hidden layer nodes Maxh allowed by the currently constructed RBF network be the number of input training samples *M*. The minimum number of nodes is set to 1. Let *L* = 1 : 1 : Maxh, that is, to search within the allowable range of the number of nodes with a step size of 1. When searching, one data is randomly selected in the input sample *c* ∈ *T*^*m*×*M*^ as the data center {*v*_1_, *v*_2_, *v*_3_}, which satisfies the

(4) $$\begin{array}{c} v_{o}=c_{\text{Round}\left(1+\mathrm{rand}*\left(M-1\right)\right)}\left(o=1,2,\cdots ,l,c={\left[c_{1},c_{2},\cdots ,c_{m}\right]}^{Y}\in T^{m\times M},l=1:\text{Maxh}\right) \end{array}$$

In Formula (4), Round(·) is the rounding function, rand is a uniform random number in the interval [0, 1], and *m* is the dimension of the input data. After determining the data center, the width of all hidden layer basis functions is set to be fixed, and the basis function expansion constant *δ* is selected according to Formula (5) to ensure that the basis functions are neither too sharp nor too smooth.

(5) $$\begin{array}{c} \delta =\frac{\max\left(\left\|v_{o}-v_{k}\right\|\right)}{\sqrt{2l}}\left(o,k=1,2,\cdots ,l,l=1:\text{Maxh}\right). \end{array}$$

After determining the center and expansion constant, the pseudo-inverse matrix method (The concept of the inverse of a square, the invertible matrix is generalized to arbitrary matrices by the pseudo-inverse of an *m* by *n* matrix *A*. Concerning *A*, the singular value decomposition (SVD) can be used to express the pseudo-inverse) is used to determine the linear parameters of the output layer of the network as follows:

(6) $$\begin{array}{c} He+q=a\Rightarrow \left[e,q\right]={\left[H,O_{M}^{\prime }\right]}^{+}\times q\left(e\in T^{l\times n},q\in T^{n}\Rightarrow \left[e,q\right]\in T^{\left(l+1\right)\times n}\right), \end{array}$$

(7) $$\begin{array}{c} \left.H\in T^{M\times l},O_{M}^{\prime }\in T^{M\times 1}\Rightarrow \left[H,O_{M}^{\prime }\right]\in T^{\left(l+1\right)\times n},a\in T^{M\times n}\right). \end{array}$$

In Formula (6), *a* ∈ *T*^*M*×*n*^ is the *n*-dimensional expected response vector of *M* training data sets; [*H*, *O*_*M*_′]^+^ is the pseudo-inverse matrix of matrix [*H*, *O*_*M*_′], of which *O*_*M*_′ ∈ *T*^*M*×1^ is an *M*-dimensional column vector whose element is 1, and *H* ∈ *T*^*M*×*l*^ is defined.

After determining the center and expansion constant, the pseudo-inverse matrix method is used to determine the linear parameters of the output layer of the network as follows:

(8) $$\begin{array}{c} H=\left\{h_{ok}=\exp\frac{{\left\|c_{k}-v_{o}\right\|}^{2}}{2\varsigma^{2}},k=1,2,\cdots ,M,o=1,2,\cdots ,l\right\}. \end{array}$$

In Formula (8), *c*_*k*_ is the *k*-th input vector of the input training data set, and *M* is the number of training samples. According to Formula (4) and Formula (8), the RBF network of this stage is constructed. Observing the output error *ϑ* of the network when l takes different values in the search space of *k* = 1 : Maxh. The value of l when *ϑ* ≤ *λϑ* is the number *k* of hidden layer nodes of the network RBF determined at this stage, where *λϑ* is the specified upper limit of error.

The first stage is the process of extracting vaccines, and the output vaccine is the number of nodes *j* = *l* in the hidden layer of the network.

Level 2: vaccination and using an immune algorithm to construct RBFNN hidden layers. An RBF network's hidden layer is nonlinear, while its output layer is linear. The Euclidean norm (distance) between the input vector and the center of the unit is computed by the argument of the activation function of each hidden unit in the RBF network.

The vaccine injected in the second stage is the vaccine *h* extracted in the first stage; that is, based on determining the network structure, the parameter *ϖ*_2_ = {*v*_*o*_, *δ*_*o*_} of the nonlinear neuron in the hidden layer is determined by learning. The details are as follows:

Antigen: the objective function to be solved by the RBFNN.

Antibody: antibody population is *S* = {*s*_1_, *s*_2_, ⋯, *s*_*N*_}, and *N* is the size of the antibody population. Any one of the antibodies is designed in the form of *s*_*o*_ = [*v*, *δ*], which corresponds to the hidden layer parameters of the RBF network. Among them, *v* = {*v*_1_, *v*_2_, ⋯, *v*_*j*_} corresponds to the data center of the hidden layer, and *δ* = {*δ*_1_, *δ*_2_, ⋯, *δ*_*j*_} corresponds to the hidden layer expansion constant. Antibodies are encoded in real numbers.

When initializing the antibody group, the vector *v* is generated by randomly selecting *j* data in the input sample *c* ∈ *T*^*m*×*M*^, and the vector *δ* is randomly generated within its value range [*f*, *i*], as shown in

(9) $$\begin{array}{c} v_{1\sim k}=c_{Round\left(1+\mathrm{rand}*\left(M-1\right)\right)}\left(c={\left[c_{1},c_{2},\cdots ,c_{m}\right]}^{Y}\in T^{m\times M}\right., \end{array}$$

(10) $$\begin{array}{c} \delta_{1\sim k}=f+\mathrm{rand}*\left(i-f\right). \end{array}$$

In Formula (9) and Formula (10), Round(·) and rand have the same meanings as Formula (4).

Antibody-antigen affinity: using the output error function of the constructed RBF network to evaluate the antibody-antigen affinity.

(11) $$\begin{array}{c} g=\overset{M}{\underset{y=1}{\sum }}\overset{j}{\underset{o=1}{\sum }}{\left(U_{o}\left(y\right)-A_{o}\left(y\right)\right)}^{2}. \end{array}$$

In Formula (11), *U*_*o*_(*y*) and *A*_*o*_(*y*) are the actual output and expected output of the *o*-th node in the *y*-th input pattern, respectively. *M* and *j* are the number of input samples and the number of hidden layer nodes, respectively.

Clonal selection: by using the clonal selection operator to generate a new generation of antibody populations, mainly including antibody cloning, mutation, and clonal selection process. When an antigen comes into contact with the immune system, its epitopes eventually only react with B-lymphocytes that have more-or-less compatible B-cell receptors on their surface, activating those B-lymphocytes. Clonal selection is the name given to this process. A single antibody is expanded into a subantibody population after cloning. The cloned subantibody group is subjected to mutation operation according to the mutation probability *a*_*n*_. The vector *v* representing the center and the vector *δ* representing the expansion constant in the antibody are mutated according to Formula (12), and Formula (14), respectively, wherein the same parameters have the same meaning as above. Clonal selection is based on affinity selection in the subantibody population after clonal mutation to retain the optimal antibody with the smallest affinity (i.e., the smallest error in the output of the hidden layer of the network).

(12) $$\begin{array}{c} v⟶v:v_{o}=\varepsilon_{1}v_{o}+\varepsilon_{2}c_{t1}+\varepsilon_{3}c_{t2}a\leq a_{n}, \end{array}$$

(13) $$\begin{array}{c} o=Round\left(1+\mathrm{rand}*\left(j-1\right)\right),t1,t2=\left(1+\mathrm{rand}*\left(M-1\right)\right),\varepsilon_{1-3}\in \left[0,1\right], \end{array}$$

(14) $$\begin{array}{c} \delta ⟶\delta :\delta_{\left(Round\left(1+\mathrm{rand}*\left(j-1\right)\right)\right.}=f+\mathrm{rand}*\left(i-f\right)a\leq a_{n} \end{array}$$

The output of the second stage is the optimal antibody in the previous generation ICSA antibody population, which is the learning process of the artificial immune algorithm after vaccination. The output is the center *v*_*o*_ and expansion constant *δ*_*o*_ of the hidden layer neurons of the RBFNN.

The third stage: the output layer of the RBFNN is constructed based on the *ϖ*_2_ calculated by the first stage and the second stage, that is, based on the matrix equation

(15) $$\begin{array}{c} Fe+q=a \end{array}$$

The network output parameters *ϖ*_3_ = {*e*_*o*_, *q*} is estimated by using the least squares method. In Formula (15), the definition of *H* ∈ *T*^*M*×*j*^ is the same as that of Formula (8), and the meaning of *a* ∈ *T*^*M*×*n*^ is the same as that of Formula (8).

The basic flow of this three-stage learning algorithm for RBFNN is shown in Figure 7, where the stopping condition is set to evolve to the maximum algebra or satisfy the desired error criterion.

## 3. Experiment on the Effect of Compound Microecological Preparation on Chicks

In this section, we discuss the experimental setup in detail.

### 3.1. Experimental Design

Numerous studies have shown the emergence of antibiotic resistance and immunosuppression in farm animals and poultry. Reduced immunity is a condition known as immunosuppression. Cell immunity and/or humoral (antibodies) immunity may be compromised. Immunosuppression can be brought on by pathogens, an unbalanced diet (deficiencies), a lack of biosecurity, poor management (stress), or a combination of these factors. It can be seen that the use of compound microecological preparations instead of antibiotics, on the one hand, improves the economic benefits of animal husbandry. On the other hand, it prevents the toxic side effects caused by drugs and has unique social and economic benefits. Studies have shown that this preparation can increase the number of T cells in the immune organs of chicks and can improve daily weight gain and meat-to-feed ratio. The identification of foreign substances by various types of immunocompetent cells is the most complex aspect of the immune system seen in vertebrates. Birds are the first vertebrate species in which a distinct lymphoid system dichotomy has been identified as follows: (1) T lymphocytes from the thymus, which act as effector cells in cell-mediated immunity, and (2) bursa-derived (b) lymphocytes, which are the precursor cells of the plasma cell that synthesizes antibodies.

In this paper, microecological compound preparations were used to feed chickens to investigate their effects on the growth performance and immune function of chickens.

Selecting normally fed day-old chicks and observing for 3 days. After culling sick and weak chickens, 200 healthy chickens with similar body weights were randomly divided into the control group and experimental group, with 100 in each group (20 in each cage, 5 cages in total). All laying hens were fed and watered ad libitum during the week and vaccinated against avian influenza with eye and nose drops. A variety of other birds, including domestic poultry, can contract the viral infection known as avian influenza. Shorebirds and wild waterfowl are frequently asymptomatic carriers. Low pathogenicity strains commonly cause respiratory symptoms in poultry. The experiment lasted for 6 weeks, and other feeding methods strictly followed the feeding methods of chickens (0-6 weeks old).

The measurement indicators are as follows: Control group: basal diet; and experimental group: basal diet +200 mg/kg compound probiotics.

The specific data is shown in Table 1.

### 3.2. Growth Performance

All chickens were weighed on the morning of the first day of the test period at weeks 0, 1, 2, 3, 4, 5, and 6 to calculate weekly gain, feed consumption, and feed weight ratio.

### 3.3. Immune Organ Index

On the 3rd, 4th, and 6th week of the experiment, 6 chickens were randomly selected. The jugular vein was incised, the spleen, thymus, and bursa were separated, blood was collected, and fat was removed to measure fresh weight and calculate the immune organ index. Jugular veins are simple to spot because they are located just below the skin. Considering that they deliver oxygenated blood to the brain. The carotid arteries are frequently visible on the surface of the neck muscle, close to the head, in chickens, geese, and guinea fowl. The chicken spleen, which is the largest peripheral lymphoid organ, is important for both bacterial and viral immune responses to acquired antigens. The bursa of Fabricius is a chestnut-sized, sac-like organ in the chicken that is anterior to the sacrum, and dorsal to the rectum. It connects to the posterior part of the cloaca via a short duct. The chicken thymus is made up of several lobes that span almost the entire length of the neck above the jugular vein on either side. The thyroid is located right next to the posterior lobe.

### 3.4. Determination of Biochemical Blood Indicators

On the morning of the first day of the 3rd, 4th, and 6th week of the experiment, 10 chickens were randomly selected every day. The cardiac blood was collected to prepare heparin anticoagulation and sterile serum samples to determine the required values. Heparin is a drug and a naturally occurring glycosaminoglycan that is also referred to as unfractionated heparin. Heparins are classified as anticoagulants because they rely on the activity of antithrombin. It is specifically used to treat unstable angina and heart attacks.

### 3.5. The Number of Intestinal Flora

Three chickens of 2, 4, and 6 weeks of age were randomly selected, then fasted for 12 hours (without water) and weighed, and the chickens were euthanized by intracardiac air injection. Colony counts were counted after 48 hours of anaerobic culture in a 37°C biochemical incubator, while E. coli was counted after 24 hours of aerobic culture in red methylene blue agar medium. Colony counts were expressed as the logarithm of the total number of bacterial colonies per gram of intestinal content [(1 gCFU)/g].

### 3.6. Plasma Total Antioxidant Capacity (T-AOC)

6 chickens of 2, 3, 4, and 5 weeks of age were randomly selected for each repetition, then fasted for 12 hours (without drinking water). The blood was collected from the fin vein, and the plasma was centrifuged at 3000 r/min for 10 minutes.

## 4. Results

In this section, we will discuss the influence on growth performance, the influence of the immune organ index, the influence of blood biochemical indicators, the influence of the number of chickens' cecal flora, and the influence of antioxidant capacity in detail.

### 4.1. Influence on Growth Performance

As can be seen from Figure 8, during the experimental period, the experimental group had a significant difference in weekly weight gain compared with the control group (*p* < 0.05) (Figure 8(a)). The weight gain of the experimental group added with the compound probiotics was significantly higher than that of the control group, and the experimental group was 15.70% higher than the control group at the age of 6 weeks. In terms of feed consumption, the ratio of the experimental group was lower than that of the control group, and the difference was significant (*p* < 0.05) (Figure 8(b)). In terms of feed-to-weight ratio, the ratio of the experimental group was lower than that of the control group, and the difference was significant (*p* < 0.05). The feed ratio of the 6-week-old experimental group was 30.37% lower than that of the control group (Figure 8(c)).

### 4.2. Influence of Immune Organ Index

It can be seen from Figure 9 that the indexes of the spleen (Figure 9(a)), bursa (Figure 9(b)), and thymus (Figure 9(c)) of the chickens in the test group were higher than those in the control group. At 6 weeks of age, the spleen, bursa, and thymus indexes of the chickens in the experimental group were 63.02%, 38.77%, and 26.82% higher, respectively, with significant differences (*p* < 0.05). The immune level of chickens is affected by the developmental status of immune organs. The increase in the relative weight of immune organs means that the immune level of the body also increases.

### 4.3. Influence of Blood Biochemical Indicators

It can be seen from Figure 10 that the total protein value of the experimental group was higher than that of the control group, and the difference was significant (*p* < 0.05) (Figure 10(a)). Regarding the blood glucose value, the difference between the control group and the test group was not significant (*p* > 0.05) (Figure 10(b)). Compared with the control group, cholesterol in the experimental group was significantly decreased (*p* < 0.05) (Figure 10(c)). The glutamic oxalacetic transaminase was significantly increased (*p* < 0.05) (Figure 10(d)), and glutamic-pyruvic transaminase was significantly decreased (*p* < 0.05). 0.05) (Figure 10(e)), and cholinesterase was significantly increased (*p* < 0.05) (Figure 10(f)). The above indicators all indicate that the probiotic compound microecological preparation has a promoting effect on the immunity of the body.

### 4.4. Influence of the Number of Chicken Cecal Flora

Around 400 to 500 different species of bacteria from 190 different genera are found in the colon of a healthy adult, but only a few of these genera together make up the majority of the feces' cultivable flora. It can be seen from Table 2 that at 2, 4, and 6 weeks of age, the number of lactobacillus cecum in the test group was slightly higher than that in the control group, indicating that the addition of the compound probiotic (Living microorganisms known as probiotics may aid in the treatment and prevention of certain diseases when consumed. The gut microbiota, a bacterial colony, plays a role in digestion, immune health, and other processes. Microbes are a class of creatures made up of bacteria, fungi, viruses, and protozoa) and its adjuvant has the potential to promote the reproduction of lactobacillus caeca. The addition of microbial complex and its adjuvant did not improve the results, and there was no significant difference in the number of *Escherichia coli* (E. coli is present in all types of poultry. In the majority of animals, including poultry, the gut naturally contains the Escherichia bacteria. Other bacteria in the gut normally keep it in check, but if large colonies form, it can result in serious discomfort, illness, and even death) between the chicken groups (*p* > 0.05).

### 4.5. Influence of Antioxidant Capacity

As can be seen from Table 3, the total antioxidant capacity of chicken plasma in the experimental group was slightly higher than that in the control group during the entire experimental period. The addition of microbial complex and its adjuvant significantly improved the total antioxidant capacity (Total antioxidant capacity (TAC) is a commonly used analyte to evaluate the antioxidant status of biological samples and can assess the antioxidant defense against free radicals produced in a particular disease) of broiler plasma (*p* < 0.05), and the experimental group was significantly higher than the control group (*p* < 0.05). This means that the addition of complex probiotics and their auxiliary substances can effectively increase the level of antioxidants in the body.

## 5. Conclusion and Future Work

This paper provided a theoretical basis for the possibility of adding probiotic complexes to chicken diets by measuring the effects of probiotic complex probiotics on growth performance, immune function, cecal flora numbers, and antioxidant capacity. When chickens were fed the prepared probiotic complex probiotic, the number of activated T cells and serum erythrocyte immunomodulatory factor activity were significantly increased. This indicated that the complex probiotics support the growth and immune function of chickens. However, there are still deficiencies in the test. This test only discussed the effect of compound probiotics on the growth and immunity of chicks. However, the optimum amount of addition in production practice and the possible effects are still unknown. Therefore, the research should continue.

## Figures and Tables

**Figure 1:** Immune hierarchy diagram.

**Figure 2:** Mechanisms of innate and adaptive immune interactions.

**Figure 3:** Principle of immune feedback.

**Figure 4:** The Process of immune memory cell formation.

**Figure 5:** Common learning methods for RBFNN.

**Figure 6:** Three-level learning structure of RBFNN.

**Figure 7:** Three-level algorithm of RBFNN based on immune mechanism.

**Figure 8:** Mean weight gain, feed consumption, and feed-to-weight ratio (g) of chicks at different stages.

**Figure 9:** Chicken immune organ index in each group (mg. g^−1^).

**Figure 10:** Effects of compound probiotic microecological additives on blood biochemical indexes of chicks.

**Table 1:** Basal diet composition and nutritional standards.

Nutritional composition	0 ~ 3 weeks (%)	4 ~ 6 weeks (%)	Nutritional level	0 ~ 3 weeks (%)	4 ~ 6 weeks (%)
Corn	63.75	60.9	Metabolizable energy (MJ/kg)	12.90	12.80
Soybean meal	25.34	28.5	Crude protein (%)	9.00	21.20
Cottonseed meal	2.88	0	Arginine (%)	0.70	1.16
Corn protein flour	1.3	1.4	Methionine+ Optine (%)	0.80	0.90
Fish meal	1.2	2.8	Calcium (%)	0.68	0.43
Wheat flakes	0.3	1.1	Total phosphorus (%)	0.41	1.10
Stone powder	0	0.1	Available phosphorus	0.95	0.71
Calcium hydrogen phosphate	1.42	1.5			
Salt	0.24	0.9			
Choline chloride	0.12	0.1			
Sodium sulfate	0.12	0.14			
Methionine	0.06	0.9			
Lysine	0.13	0.12			
Soybean oil	1.9	0.04			
Vitamins	0.04	0.3			
Premix	1.2	1.2			
Total	100	100			

**Table 2:** Effects on the numbers of chicken cecum and *Escherichia coli*.

Project	Week age	Control group	Test group
Lactic acid bacteria	2	7.93	8.88
	4	8.57	8.95
	6	8.04	8.13

*Escherichia coli*	2	8.08	7.60
	4	8.17	7.84
	6	8.55	8.28

**Table 3:** Effects on total antioxidant capacity of chicken plasma.

Week age	Control group	Test group
2	23.01	24.91
3	14.98	19.55
4	17.06	20.39
5	17.39	22.02

## Data Availability

No data were used to support this study.
